# Deep-Learning-Based 3D Reconstruction: A Review and Applications

**DOI:** 10.1155/2022/3458717

**Published:** 2022-09-15

**Authors:** Yinhai Li, Fei Wang, Xinhua Hu

**Affiliations:** ^1^College of Mechanical and Electrical Engineering, Jinhua Polytechnic, Jinhua 321007, Zhejiang, China; ^2^Key Laboratory of Crop Harvesting Equipment Technology of Zhejiang Province, Jinhua Polytechnic, Jinhua 321007, Zhejiang, China; ^3^College of Creative Arts, Jinhua Polytechnic, Jinhua 321007, Zhejiang, China

## Abstract

In recent years, deep learning models have been widely used in 3D reconstruction fields and have made remarkable progress. How to stimulate deep academic interest to effectively manage the explosive augmentation of 3D models has been a research hotspot. This work shows mainstream 3D model retrieval algorithm programs based on deep learning currently developed remotely, and further subdivides their advantages and disadvantages according to the behavior evaluation of the algorithm programs obtained by trial. According to other restoration applications, the main 3D model retrieval algorithms can be divided into two categories: (1) 3D standard restoration methods supported by the model, i.e., both the restored object and the recalled object are 3D models. It can be further divided into voxel-based, point coloring-based, and appearance-based methods, and (2) cross-domain 3D model recovery methods supported by 2D replicas, that is, the retrieval motivation is 2D images, and the recovery appearance is 3D models, including retrieval methods supported by 2D display, 2D depiction-based realistic replication and 3D mold recovery methods. Finally, the work proposed novel 3D fashion retrieval algorithms supported by deep science that are analyzed and ventilated, and the unaccustomed directions of future development are prospected.

## 1. Introduction

With the development of 3D modeling technology and data processor graphics, 3D standards have been widely customized in CAD, VR/AR, and autonomous trends. At the same time, the long-term update of technologies such as 3D reconstruction and 3D typesetting has also made the process of procreate 3D fork easier. Due to the tragic increase in 3D execution enumeration, orientation of the fashion database and renovation and prenominal of pattern cannot be done manually. In the orchestration of the recurrent accord of the obedient, the 3D model of each province has its own proceeding database management system and agreed redintegration techniques.

Efficient and critical recovery and management has attracted more and more researchers [1–13]. Although message-based search engines are very common, for high-dimensional data such as 3D models, it is stubborn to use textual information to summarize the size of the data. Secondly, the textbook information of drivers in various fields is prone to errors and failures due to differences in speech, training, and professional attire. Retrieving a 3D plan for full realism with only text or prompts is laborious. The designed 3D sample recovery technology can accurately restore and match the 3D model [1], that is, the design conforms to the teaching of the 3D model itself. In the model-based 3D mode recovery process, when processing 3D shape data, it is necessary to first extract the form from the standard and convert the 3D model into various configurations of 3D virtual feature descriptors.

3D fashion renewal methods are divided into three categories: voxel-supported methods, peculiarity-color-supported methods, and scene-based methods. Voxel uphold is used. Both methods [3] and peculiarity loss-supported regularity [5] are used after extracting the exalted-system complete suit of the 3D model by build the suiting feature extraction mesh on the pristine 3D design. Appearance-supported methods [6, 9] use a substantial camera to render a 3D model and use the hold determine of 2D conception to delineate the original 3D design. Concept-based algorithms for 3D models also implement class problems due to the digestion technique of unmixed letters in 2D image processing. Despite the religious significance of design-supported 3D fashion restoration methods, the acquisition and annotation of complete 3D fashion movements remains an underdeveloped effort. With the development of non-hybrid neural networks and the development of a large number of 2D display datasets, the classification and recognition techniques of 2D images have been well established. Learning from 3D Appearance for Relevant Notification and Support 3D fashion is also a pressing issue in the modern donkey era [10(2)]. 2D shows supported 3D mold recovery modes, i.e., the recovery prospect is 2D appearance and the recovery slice is the 3D model. According to the different representations of the 2D picture, algorithms can be digitated into two categories: methods supported by 2D real images and methods supported by 2D designs. The way based on 2D real images [11] is to drop the form on the kerçek image, and the image rise is a photo taken at regular intervals. The 2D contour support method [12] extracts shapes from known sketches. Compared to model-supported 3D model retrieval methods, 2D image-based 3D mold restoration methods appear to be more problematic in terms of shape twinning (prenominal), but are easier to own and more widely used in the name of restoration display. In this paper, the 3D model restoration algorithms of the modern donkey era are synthesized firstly, and then different 3D plan restoration algorithms are classified according to the different 3D model retrieval tasks, and the algorithms under each type are psychologically analyzed. Among them, this note focuses on analyzing the strengths and weaknesses of 3D examples in other representations, such as voxels, stage clouds, and views of standard supported 3D model recovery algorithms. Aiming at the cross-domain 3D model recovery algorithm program based on 2D kerçek portraits, this paper defines the scenarios where the 3D fork does not contain categories, and focuses on analyzing the performance of unsupervised grant learning in unsupervised disaster-ruled 3D dummy recovery. For contour-based 3D floor plan retrieval algorithms, this paper focuses on lateral empire retrieval and twinning of 2D sketches and 3D models under giant modal competitions. Finally, this paper analyzes and summarizes the existing problems of 3D fashion retrieval algorithm rules, and discusses prospects in the new development direction in this field, which provides new ideas for replication and deliberation in this field.

In this note, filter abundance images and articulated 3D feature blackening data are used to discover channel flatness through a neural network. For non-planar parts, a custom 3D network classifies and detects the type of outer end. The proof is first illuminated by structured light. From the outside of the road, the depth appearance of the runway is calm, and the performance is more tense and clear for perception. The periphery of the ruined lane is dodged, the foreign object feature cloud extraction is carried out on an uneven route, and the sporadic details of the docking details such as similitude and experimental experience show that after adaptive settlement for the concave and reflectivity of different pavements, the alien motivation on the runway can be effectively detected.

## 2. Related Work

In recent years, with the rapid development of fuzzy neural networks and the advent of comprehensively decentralized 3D model datasets, deep science methods have been tailored [10–19]. The learning and representation of 3D models has become a common survey rule in 3D planar survey processing. Similar forms of 3D standards include voxel, point sully, and views, so at this stage, according to the different representations of 3D shape, the research described can be roughly divided into voxel-supported, moment cloud-based, opinion-based, and hybrid 3D model restoration methods.. Voxel-based 3D bifurcation recovery methods typically use crude and systematic 3D meshes to example 3D designs, and perform 3D volume and pooling operations on them to refer to higher-order features to learn representations. Qi et al. [13] discussed a Multi-Orientation Voxel Convolutional Neural Network (MO-VCNN) that uses a weight-assigned 3D Convolutional Neural Network to obtain 3D voxel features in different orientations. Then a max pooling operation is performed to stack the features, and finally the form of the stack is input into another 3D convolutional plexus for prediction and good inference. To reduce computational cost and improve effectiveness, Li et al. [14] discusses the use of room detection filters, which are adaptively distributed in a three-dimensional space by learning to change the adjustment of the discovery filters. Instantaneous staining-supported 3D model recovery means attracting 3D coordinate samples from the 3D dummy surface to form 3D point sets for learning demonstrations. The objects of the 3D stage shine in the unstructured and irregularities of the project factory. Klokov et al. talk about a k-D meshwork, which first uses a k-dimensional tree (k-D wood) to represent stage blacken, and then processes the point cloud according to the data structure. Inspired by the suit twinning algorithm [15], Xie et al. proposed a selfish attention model used to design the shape of special stains according to the context. View-based 3D pattern retrieval methods typically provide each 3D sample with a clot of a 2D foreground image, and then use a 2D convolutional neural network to extract relevant features. According to Bai et al., Hausdorff distances between consent survey sets were analyzed and a view-based 3D fork recovery system, GIFT, was designed. Su et al. [6] proposed a multi-scene convolutional neural network (MVCNN), which is first interested in cutting convolutional plexuses to extract forms from view replicas, and then performs max-pooling on the view dimension to aggregate shapes.. However, since the grid discards non-maxima in the max-pooling operation, it may not be able to exploit multi-view features maturely. In response to this deficiency, Wang et al. proposed a view group and pooling algorithm based on the judgment of the advantage set, and performed the pooling transaction operation after the multi-view determination, and maintained a good experimental effect. Other scholars have demonstrated that Long Defect Prescription Recall (LSTM) can be employed to aggregate features from multiple survey appearances; in addition, Chen et al. proposed a design that uses a iterate attention standard to automatically choice a view extend to carefully identify 3D endeavors. converse a Panoramic Convolutional Neural Network (PANORAMA-supported CNN, PANORAMA-CNN) that uses the obstacles of a panorama-supported convolutional nerval network to teach relate 3D conceit. Hybrid methods comprehensively relate to the representation of two or more 3D dummies of bony progress. According to Lu et al., the proof analyzes the relationship between the model form and scene form in 3D models. You stay. proposed a moment-table related network (PVR-Net) to liquefy indicate cloud features and manifold survey systems, and realize exact events. Reference 26 uses FusionNet to unite 3D sketch supported on a voxel shape and perception features for 3D dummy acknowledgment and restoration. Demonstrates digesting the intensity delineate and hiding the mappemonde of the 3D intend to ameliorate the utterance expressing the 3D illustrate.

Image-supported 3D virtual restoration is also an optional research judgment in the augmentation of fashion-based 3D example restoration methods. The 3D fork recovery course supported on 2D images, i.e. the retrieval object is a 2D image, the retrieval object is a 3D fork, and the 2D image and the 3D pattern are the same.

The modal difference between the criteria poses a big problem for 3D bifurcation retrieval. According to the different representations of 2D images, algorithms can be divided into two categories: methods supported by 2D true images and methods supported by 2D contours. Among the 3D model retrieval methods supported by a 2D realist cast, the unsupervised oblique-realm 3D bifurcation recovery method has attracted the attention of many researchers. For retrieval and identification dummy, Zhou et al., [10] proposed a two-layer enlay alignment network (DLEA) that jointly enforces the discipline of the model using an adversarial domain bounding algorithm and class center alignment. Li et al. [11] talk about a multi-perspective and multi-distribution academic approach. Data acquisition and related processes learn by learning two coupled subspaces that map the source domain shape and target region features to the usual domains. Domain Adversarial Neural Grid (DANN) employs an adversarial domain design algorithm to align source domain data with slice domain data. A hurdle for sketch-supported 3D model retrieval methods is addressing the large formal differences between 2D designs and 3D patterns. Zhu et al. proposed to use a trial domain neural network (CDNN) to narrow the difference between 2D depictions and 3D shapes. Dallas et al. designed a 3D fork retrieval system to assist multimedia query. The system extends the 3D model to the determination of 2D similarity and resolves the similarity between other models by referencing the shape of the 2D appearance.. applies the Bag-of-Feature (BoF) approach which is inferior to 3D model restoration in 2D electronic computer vision. In addition, Eitz et al., proposed combined BoF and Gabor Provincial Flax Support Feature (GALIF) for a sketch-based 3D plan restoration survey. Besides the BoF coding algorithm, Local Constrained Linear Coding (LLC) is another summarization method widely used in image classification, which preserves the topical features of images. Biasotti et al. proposed a Busy LLC method for 3D shape recovery. In addition, Xie et al. collected valid forms from different 2D projections of 3D models. Tasse proposes a new cross-empire retrieval approach, which embeds the attempts of different modalities into semantic feature vectors to obtain feature knowledge.

Voxel-based methods exploit the aggregation of voxels within a 3D time segment to represent 3D patterns, and then rely on neural networks on a voxel basis. Character extraction forms and enables 3D shape recognition and recovery. The 3D ShapeNets network proposed by Wu et al. [3] uses confidence distributions of binary variables on a 3D voxel grid to represent 3D geometric models. For each 3D design, build a 30 × 30 × 30 3D grid, delineating each 3D grid as a binarized vector: meaning the voxel is inside the mesh, 0 means the voxel is not inside the mesh. 3D ShapeNets proposes a deep convolutional network for teaching voxelized shapes of 3D stencils in 3D meshes. The mesh structure has a total of 5 cluster structures: the first convolutional layer has 48 convolution kernels, and each convolutional layer has 48 convolution kernels. The kernel greatness is 6, the convolution gait is 2; the other convolution base has 160 convolution kernels, each convolution kernel size is 5, and the twist straddle is 2; the third convolution layer has 512, each. The size of the vortex core is 4; the fourth layer is the fully connected belt of 1200 secrets; the ⅕ layer is the last sofa with 4000 hidden units, the output of this sofa is used as the full feature of the 3D dummy. Voxel-backed 3D shape processing algorithms renormalize 3D models, and 3D convolutional neural networks can be used for feature learning. A 30 × 30 × 30 grid requires many parameters in a neural network that has 6 2D appearances of 165 px × 165 px, but accounts and commemorates the amount of consumption wax with the fortitude of the third command, so the 3D ShapeNets plexure composition performs poorly on higher resolution 3D standard datasets.

Local feature aggregation is a very familiar and well-established approach when considering 2D images or 3D floor plans. Recently, thinkers discovered that extinction-to-termination deep 3D convolutional neural networks (3D-deep CNN, 3D-DCNN) achieve good reasoning in classification and retrieval tasks of 3D models [3]. However, 3D-DCNN-based methods have obtained useful problems. There are also shortcomings: on the one hand, it lacks invariance to 3D rotation, and on the other hand, the design quantification is too rough during touch and lacks detailed geometric features. Furuya et al. proposed a complete local feature aggregation mesh DLAN. The network construction can be divided into a singing form extraction model and a form aggregation module. The local feature aggregation model extracts and encodes cross-sectional 3D features and generates intermediate direct local shapes using 3D convolutional seams and perfectly correlated layers. The feature aggregation module collects regional 3D features, and the mid-level topic feature Embarrass calculated by the local form extraction module is a simple form of each 3D model by pooling the boost. Finally, enrichment-connection boosting can be used to suppress or condense ubiquitous features, and the final features are used for 3D model retrieval.

The key to the identification of moment damage data docking is to select the data points reflecting the geometric characteristics of the target from the spatially diverse data information for feature identification. The unmixed letter technique has been applied to fields such as feature genealogy, speech recognition, and electronic computer vision after the new fast unraveling that is widely used. Deep science uses shape descent [7] and teaches deep labelling shapes through several levels of nonlinear mapping, which is consistent for formal learning under ensemble data, and convolutional neural networks (CNN) are a typical one which can handle several ft. convolution, pooling, etc. operate on the data, and gradually refer to features from the shoal to generalize [8], which can effectively extract the secret features of high-dimensional data. At the same time, its unparalleled network configuration can effectively weaken the enumeration of parameters, reduce the complexity of the model, and facilitate the education and requirements of the model. This article attempts to use Convolutional Neural Networks. The spatial-territorial analogy (spatial-local relationship) consists of various types of data. Correctness is not limited by the way the data are represented. For data such as pictures that can be represented in an ordered domain, the volute operator has been shown to be effective in exploring such correlations, and CNNs have been successful on a variety of tasks for data whose extent is smaller than the extent of the ambient space (such as faces) in all docking categories in 3D rove or 2D room), if these data are represented as point clouds in the surrounding space, and if not a coarse grid of the entire track, then the result will be a uniform reformation. However, the guided way that the distortion loses its influence on the features will make it difficult for the convolution operator to exploit the spatial correlation between stage impairments [9].

In a symmetric mesh, each mesh cell is associated with a feature. In staged damage, spines are sampled from local neighbors, similar to local points in a system grid, and each detail is associated with a feature, an ordinal point, and its coordinates. However, due to the lack of a regular grid, it is difficult to detect details in the specification command. Suppose we use the same twist kernel as in the equation. The order given by the regular grid construction constrains a proper learning execution, the details are sampled from territorial neighbors and can therefore be in any direction. Through the same volume action, the three-dimensional space of the point cloud defines the point cloud images of all scales at the end, which helps to further explore the spatial characteristics of the object. In order to better achieve classification and division, the layers are combined. The thorn-dirty features of different scales in space can fully mine the existence information of the target and identify the blackening of details more effectively. The realization of this goal is a drastic division into two projections. First, non-uniform downsampling corrects the organic features of the object, and spatial feature learning is performed for each specific impairment to obtain the shape of each management; then these regional features in different directions are combined to obtain multiple spaces containing rich instructions feature and learn it using a convolutional neural network.

The neural cobwebs used in the experience first convert input points (target instants or pavement points) through a four-top space-warping web into fewer morphological instants, but each morphological point contains richer spatial information, and then pass through a four-top space-warping web. The full intersection occurs after the layer, and the point cloud data are digitized into 4 categories by a layer of 4 full constants, namely nigger, nut, indeterminate appearance, and no separation object. Although blurred remote objects cannot be effectively identified for partially segmented foreign objects after projection interception, no foreign objects can be clearly distinguished, and Reticulum finally calculates the credibility of several data through the Softmax layer. ModelNet40 data adjustment is used to evaluate the classification effect and recovery performance of the above scheme, and the ShapeNet Core55 data set is used to evaluate the retrieval effect of the above algorithm. Both the ModelNet40 dataset and the ShapeNet Core55 dataset provide standard 3D obj reformatted lines that can be regenerated as voxel data, point cloud data, or multi-judgment data. The number of relishes of each type in the ShapeNet Core55 dataset is not uniform. Therefore, when wearing the ShapeNet Core55 dataset to analyze the recovery behavior of the algorithm program, in order to better comprehensively evaluate the recovery events of different symbols of the standard, two methods are adopted. There are different methods for evaluating lickpot estimation: macro-average and micro-average. Macro-averaging refers to computing different recovery metrics (F, delineation, NDCG) for all samples on the entire dataset, and each 3D bifurcation example uses the same case in estimating the recovery metrics. Micro-Norma refers to the first computed recovery metrics (F, delineate, NDCG) within each type.

The restoration demor for each category is Norma, and each group provides the same assertion when predicting recovery metrics. The 3D design playbill algorithms verified by the above models all gain on a well literate archetype, adopt distinct 3D plan protrusion methods (voxel, item smear, manifold measurements), plan a forced non-hybrid network construction, and extract violent plane features for use. A 3D sample condyle model 3D mold is used for restoration or classification. 3DshapeNets voxelize 3D shape data, and each 3D pattern is represented as a 30 × 30 × 30 3D grid; DLAN first decomposes local proposals for 3D models using an average voxel grid, then stacks them around notifications; PointNet and PointNet++ It are intended to use the full Reticulum structure to temporally extract shape from point damage data; MVCNN, RotationNet, GVCNN, and View-GCN select multi-view data as input data, indicate different multi-view liquefaction methods, and extract high-order wide heuristics.

## 3. Conclusions

When restoring a 3D shape, the retrieval attempt is a 3D standard, and the problem foreground can be a 3D design or a 2D appearance. Accordingly, this paper ranks 3D plan restoration methods based on cunning learning: fork-based 3D model retrieval algorithm rules and 2Dlikeness-based 3D model restoration algorithms. According to the 3D standard retrieval algorithm rules supported by the example, this paper focused on analyzing the different display methods of the 3D floor plan: voxel support method, thorn-coloring support method, and foreground support rules, each order has certain advantages and disadvantages. 3D sample voxelization refers to the conversion of an appropriate 3D model into structured data, which can be directly processed by a 3D convolutional neural network, but the 3D voxel grid takes up too much memory, and the existing computational sway limits high separation 3D model voxelization function. The moment damage type data can characterize the 3D prongs as comprehensively as possible, but the point blackening data are unstructured and cannot be represented by a grid like a 2D image. The pose of the mold on the orbit is arbitrary, only when the object rotates in, the object itself does not change, but its three-dimensional coordinates have disappeared in a large walk. In practical application scenarios, the prick count will have a large error, and a commendable algorithm rule is essential to deal with the damage data of other scales. Although view-supported methods have been successful in preserving the deep literature of 2D portraits, they also cannot use images for each ken indefinitely due to memory constraints, and a fixed large number of views may not be efficient enough to fully exhibit stereo. At the same time, there is some redundancy in notification between each lead. In augmentation, second-hand 2D view data inevitably misses some 3D structural information, especially in practical application scenarios, when a 3D dummy is involved, it is difficult to require a fixed large number of views to thoroughly represent 3D models.. If the mastery of various 3D model representations can be fixed while reducing ad redundancy, it could be a monumental inspiration for the 3D standard prominence. Aiming at the 3D design restoration algorithm program supported by 2D images, this paper makes a preference between 2D live portraits and 2D sketches for 2D idols. Two-dimensional kerçek images have spawned a plethora of advertisements, and various obscure academic methods are exploring how to extract the rich information in portraits more exhaustively, with good results. And the 2D image data adjustment is very complete, with rich annotations and complete recommendations to practice uncertain dummies; second-hand observation give learning, infected with the real face of 2D as the source empire and 3D design as a docking field, from 2D Appearance Transferring the information book learned in 3D standards into 3D fashion has a lot of real-world implications. Therefore, this paper details an algorithmic procedure for unsupervised disappointment orbit 3D restoration that supports 2D real images. The algorithmic procedure determines that 3D models do not contain labeled spectacles and converges on the analysis of unsupervised transfer letters in 3D fashion recovery in the unsupervised trial domain performance. This nihilistic colonization of 2D idols and 3D molds is difficult to completely destroy the depth Ball Fitness Algorithm program still wins a decent trial event, and makes for a great guide party for resuming the hard work of 3D design. The 3D plane restoration algorithm rules based on 2D contours can improve the effectiveness of 3D model modeling and analysis more conveniently and intuitively in practical applications. The construction of the 3D example is very complex. The collected 3D molds can be recycled very well, which is of great help to the modelers and users of the 3D models. Based on this, this paper focuses on the peevish-domain retrieval and matching of 2D planes and 3D models under the 3D standard restoration algorithm supported by the design, and relies on deep erudition and metric learning to have certain observability. However, because the 2D depiction is too simple, the modal difference is large, and the 3D shape is hard, there are still problems in the recovery algorithm rules of the 3D model based on the depiction, which will be the focus of the next research.

## Data Availability

The data can be obtained by requesting the correspondence author.

## References

[1] Han Z., Guoqi B., Kai L. (2019). Simple calibration method for three-dimensional imaging system with structured light. *Advances in Lasers and Optoelectronics*.

[2] Turk G. The PLY polygon file format. https://blog.csdn.net/eloudy/article/details/70478083.

[3] Lin T. (2017). *Research on 3D Point Cloud Data Reduction and Compression [Master's Thesis]*.

[4] Xiao T., Chuankun L., Lening L. (2019). Research on leak detection of vinyl spherical tank based on convolutional neural network. *Safety Health and Environment*.

[5] Xiaoliang W., Chaoqun T. J. (2012). Fault diagnosis of high-speed plunger pump based on LSTM and CNN. *Journal of Aeronautics and Astronautics*.

[6] Hongbin Z. (2019). *Research on 3D Object Detection Algorithm and Labeling Tool Design Based on Point Cloud [Master's Thesis]*.

[7] Li G., Yi J., Chunping L. (2009). Three-dimensional point cloud classification method based on multimodal feature fusion. *Computer Engineering*.

[8] Jinhua Z., Jun Z. (2012). Research on foreign object detection system of airport runway. *Modern Electronic Technology*.

[9] Liu A. A., Nie W. Z., Gao Y., Su Y. T. (2018). View-based 3-D model retrieval: a benchmark. *IEEE Transactions on Cybernetics*.

[10] Zhou H., Liu A. A., Nie W. (2019). *Dual-Level Embedding Alignment Network for 2D Image-Based 3D Object Retrieval. Proceedings of the 27th ACM International Conference on Multimedia*.

[11] Li W., Liu A., Nie W. (2019). *Proceedings of EurographicsWorkshop on 3D object retrieval. [S.l.]*.

[12] Li B., Lu Y., Li C., Godil A. A. (2014). *SHREC' 14 Track: Extended Large Scale Sketch-Based 3D Shape Retrieval. Proceedings of Eurographics Workshop on 3D Object Retrieval*.

[13] Qi C. R., Su H., Niebner M., Dai A., Yan M., Guibas L. J. (2016). *Proceedings of the IEEE Conference on Computer Vision and Pattern Recognition. [S.l.]*.

[14] Li Y., Pirk S., Su H., Qi C. R., Guibas L. J. (2016). FPNN: field probing neural networks for 3D data. *Advances in Neural Information ProcessingSystems*.

[15] Belongie S., Malik J., Puzicha J. (2000). Shape context: a new descriptor for shape matching and object recognition. *Advances in Neural Information Processing Systems*.

